The article "Clinical Study of Different Treatment Methods for Tuberculous Pleuritis Complicated with Pleural Tuberculoma" was retracted in 2023. Reasons: unreliable results or conclusions; lack of ethics approval or compliance; concerns about the data; concerns about the peer review.

# Clinical Study of Different Treatment Methods for Tuberculous Pleuritis Complicated with Pleural Tuberculoma

**DOI:** 10.1155/2022/5666067

**Published:** 2022-08-27

**Authors:** Xiaoling Zhang, Jingyu Chi

**Affiliations:** Four Tuberculosis Areas, Shandong Public Health Clinical Center, Jinan, Shandong 250001, China

## Abstract

**Objective:**

To compare the clinical efficacy and adverse drug reactions of four different schemes in the treatment of pleural tuberculoma.

**Methods:**

A total of 120 patients with pleural tuberculoma admitted to the Tuberculosis Department of our hospital from January 2018 to January 2021 were selected as the research subjects. According to different treatment methods, the patients were divided into four groups, with 30 cases in each group. They were as follows: group A received classical HRZE regimen, group B received HRZE+pleural injection, group C received HZE+rifabutin, and group D received HZE+rifabutin+pleural injection. All patients were treated intensively for 3 months and then consolidated treatment for 6 months according to the patient's condition. The absorption of lesions in the four groups at different time was compared, and the occurrences of adverse drug reactions and treatment outcomes during treatment were recorded.

**Results:**

After 3 months of treatment, compared with groups A, B, and C, the number of significantly absorbed cases and effective cases in group D increased, while the number of invalid cases decreased. However, there was no statistical significance in the absorption of lesions between the four groups (*χ*^2^ = 8.272, *P* = 0.507). In addition, pairwise comparison showed no significant difference in the absorption of lesions (*P* > 0.05). After 9 months of treatment, there was no significant difference in the absorption of lesions among the four groups (*χ*^2^ = 8.795, *P* = 0.185), but the absorption of lesions in group D was significantly better than that in group A (*P* < 0.05). During treatment, the incidence of adverse reactions in the four groups was significantly different (*χ*^2^ = 8.779, *P* = 0.032). Pairwise comparison showed that the incidence of adverse reactions in groups C and D was significantly lower than that in group A (*P* < 0.05). The total treatment course of group A was 9-16 months, and 10 cases (33.33%) still had residual lesions or pleural thickening at the end of treatment. The total course of treatment in group B was 9-12 months, and 7 cases (23.33%) still had residual lesions or pleural thickening at the end of the course of treatment. The total treatment course of group C was 9-16 months, and 8 cases (26.67%) still had residual lesions or pleural thickening at the end of treatment. The total course of treatment in group D was 9-12months, and there were still 2 cases of residual lesions (6.67%) at the end of the course.

The article "Clinical Study of Different Treatment Methods for Tuberculous Pleuritis Complicated with Pleural Tuberculoma" was retracted in 2023. Reasons: unreliable results or conclusions; lack of ethics approval or compliance; concerns about the data; concerns about the peer review.

**Conclusions:**

HZE+rifabutin+pleural injection against tuberculosis therapy has a significant clinical efficacy in the treatment of pleural tuberculoma, which can more effectively improve the clinical symptoms of patients, improve the efficacy, and reduce complications, with a good prognosis, worthy of clinical promotion.

## 1. Introduction

Tuberculous pleurisy is the second most common extrapulmonary tuberculosis after lymph node tuberculosis. It accounts for about 3% to 5% of tuberculosis in the United States and can reach 30% in countries with high tuberculosis burden [1]. As a localized lesion in the pleural cavity, pleural tuberculoma can occur in the parietal pleura or visceral pleura [2] and is one of the rare clinical diseases. At present, its pathogenesis is not clear, and most scholars believe that it is a caseous mass wrapped in fibrous tissue formed by the concentration and drying of local tuberculosis tissue caused by fibrous connective tissue hyperplasia and pleural thickening and adhesion in the course of the development of exudative tuberculous pleuritis [3, 4]. Pleural tuberculoma can occur in all age groups but is generally believed to be more common in young adults. The incidence of pulmonary tuberculoma is 0.62%-5.7%. Most patients with pleural tuberculoma have definite tuberculous pleurisy or pulmonary tuberculosis (75%-96%), but a small number of patients have no definite history of tuberculosis and only find the lesions during physical examination (4.0%-25%) [5–7]. Patients with tuberculous pleuritis develop pleural tuberculoma even after regular intensive antituberculosis therapy, which is classical HRZE scheme. Clinical data show that pleural tuberculoma occurs more within 3 months of antituberculosis treatment. The clinical practice is to continue the original regimen of antituberculosis treatment, and most of pleural tuberculoma can be absorbed in 3~18 months. If the disease persists or the patient requires, surgical resection is feasible [8, 9]. In recent years, we find that more and more patients developed pleural tuberculoma in the course of treatment in clinical work. Classical antituberculosis drugs are still the preferred method for the treatment of pleural tuberculoma, but they have many adverse reactions, which sometimes aggravate or prolong the disease course of patients, leading to drug resistance of tubercle bacillus in some patients and poor prognosis [10]. Rifabutin is a semisynthetic rifamycin, similar to rifampicin, rapidly absorbed in the gastrointestinal tract, with good lipid solubility, which can be widely distributed in tissues and cells. It is well tolerated and has fewer side effects than rifampicin [11, 12]. In addition, since antituberculosis drugs are difficult to penetrate into the pleural tuberculoma lesions, the effect of chemotherapy solely relying on drugs is poor [3, 13]. On the basis of systemic antituberculosis treatment, combined with intrapleural tuberculoma injection, the drug concentration in pleural tuberculoma can be effectively increased, which is beneficial to improve the curative effect. In order to reduce complications and improve efficacy, 120 patients with pleural tuberculoma who were initially diagnosed in our hospital were treated with different treatment schemes in this study, aiming to observe the clinical efficacy of different treatment schemes and provide clinical practice for better treatment of pleural tuberculoma patients. The report is as follows.

The article "Clinical Study of Different Treatment Methods for Tuberculous Pleuritis Complicated with Pleural Tuberculoma" was retracted in 2023. Reasons: unreliable results or conclusions; lack of ethics approval or compliance; concerns about the data; concerns about the peer review.

## 2. Materials and Methods

### 2.1. Materials

A total of 120 pleural tuberculoma patients admitted to the Tuberculosis Department of our hospital from January 2018 to January 2021 were enrolled as the research subjects. Patients were randomly divided into four groups and then given different treatment regimens, 30 cases in each group. Group A was given classical HRZE regimen; group B was given HRZE+pleural cavity infusion; group C was given HZE+rifabutin; and group D was given HZE+rifabutin+pleural cavity infusion. Inclusion criteria are as follows: (1) a history of “tuberculous pleuritis,” (2) suspected pleural tuberculoma, (3) complete clinical data, (4) informed consent to the study from patients and their families, and (5) patients older than 18 years old. Exclusion criteria are as follows: (1) severely infected persons; (2) patients complicated with serious cardiovascular and cerebrovascular diseases, nephropathy, and autoimmune diseases; (3) patients complicated with malignant tumor; (4) patients complicated with cognitive and behavioral ability insufficiency; (5) pregnant or lactating women; (6) patients with drug withdrawal or change of treatment plan due to serious adverse reactions; (7) patients with previous antituberculosis treatment; and (8) patients who dropped out of the clinical study or were lost to follow-up.

### 2.2. Therapeutic Methods

All patients received general symptomatic treatment such as anti-infection, fluid rehydration, nutritional support, and correction of electrolyte disorders. On this basis, group A was given classical HRZE regimen. The drugs included isoniazid tablet (H) (Southwest Pharmaceutical Co., Ltd., SFDA approval number: H50020124, specification: 0.1 g/tablet, dosage: 3 tablets/time), rifampicin capsule (R) (Chengdu Tiantai Mount pharmaceutical Co., Ltd., SFDA approval number: H51022701 of specification: 0.15 g/tablet, dosage: 3 tablets/time), pyrazinamide tablets (Z) (Guangdong South China Pharmaceutical Group Co., Ltd. SFDA approval number: H44020761, Specification: 0.25 g/tablet, dosage: 3 tablets/time), and ethambutol tablets (E) (Guangdong South China Pharmaceutical Group Co., Ltd. SFDA approval number: H44020758, specification: 0.25 g/tablet, dosage: 3 tablets/time), all of which were administrated orally, once a day. Group B was given HRZE+pleural cavity medicine injection regimen, a joint pleural cavity medicine injection on the basis of the treatment of group A. The specific operation was as follows: the patient underwent B-ultrasound examination to determine the puncture point; the skin was sterilized; the surgeon worn sterile gloves, covered the hole drapes, and vertically inserted the needle with 0.2% lidocaine at the upper edge of the rib at the puncture point. The B-ultrasound positioning tip was located in the center of the puncture, and 0.1 g (2 mL) isoniazid was injected locally, and the needle was removed. The patient was asked to rest in bed. Group C was given HZE+rifabutin. The drugs included isoniazid+pyrazinamide+ethambutol+rifabutin. Rifabutin (Sichuan Med-Shine Pharmaceutical Co., Ltd., SFDA approval number: H2007296, specification: 0.15 g/tablet, dosage: 2 tablets/time) was administrated orally, once a day. Group D was given HZE+rifabutin+pleural infusion regimen, a joint pleural cavity medicine injection on the basis of the treatment of group C. The procedure was the same as that of group B, and patients in all four groups received intensive treatment for 3 months. If the laboratory sputum smear is still positive after 3 months of intensive treatment, the treatment would be prolonged. The four groups received the same consolidation treatment: isoniazid tablet (0.1 g/tablet) and rifampicin capsule (0.15 g/tablet), orally, three times a day, for 6 months.

The article "Clinical Study of Different Treatment Methods for Tuberculous Pleuritis Complicated with Pleural Tuberculoma" was retracted in 2023. Reasons: unreliable results or conclusions; lack of ethics approval or compliance; concerns about the data; concerns about the peer review.

### 2.3. Observational Indices

(1) Age, gender, complications, the levels of albumin (Alb), erythrocyte sedimentation rate (ESR), fasting blood glucose (FBG), and lactic dehydrogenase (LDH) were recorded at admission. (2) Chest CT scan features were recorded. (3) The location, number, and size of pleural tuberculoma were recorded. (4) Pleural tuberculoma absorption was compared among the four groups at the third month of treatment, and the actual course of treatment and the final treatment outcome of all patients were recorded. (5) Clinical cure rates of patients in four groups were recorded. (6) The incidence of adverse reactions during treatment was recorded, including skin rash, liver damage (increased alanine transaminase (ALT)), cytopenia (decreased platelets (PLT)), and renal function (increased uric acid (UA)).

### 2.4. Evaluation Criterion

The evaluation of pleural tuberculoma absorption was carried out according to the *Clinical Diagnosis and Treatment Guidelines: Tuberculosis Volume* developed by the Chinese Medical Association [14], and the outcome of pleural tuberculoma was measured and observed by chest CT scan: (1) “significantly absorbed “ refers to the complete absorption of the lesions in the lung or the reduction of the pleural tuberculoma more than 50%~80% after treatment. (2) “Effective” means the absorption of the lesion between 30% and 50%. (3) “Invalid” refers to the reduction of pleural tuberculoma in patients with less than 30% or no significant reduction. (4) “Deteriorated” refers to the trend of increasing diameter or number of pleural tuberculoma in patients. Clinical cure is as follows: complete disappearance of symptoms and signs, obvious absorption of lung lesions, and negative culture of mycobacterium tuberculosis in sputum for three consecutive times or more [15]. All patients were followed up to the end of the treatment course.

### 2.5. Statistical Analysis

SPSS 22.0 software was used for statistical analysis. Measurement data conformed to the normal distribution were expressed in the form of $\bar{x}\pm s$ and tested by independent sample *t*-test between two groups. Data not conformed to normal distribution were tested by the Mann-Whitney *U* rank-sum test. One-way ANOVA was used for comparison between multiple groups. Counting data were expressed as *n* (%), and the comparison between groups was performed by *χ*^2^ test. *P* < 0.05 indicated significant difference.

## 3. Results

### 3.1. Comparison of General Data of Patients in Four Groups

Before treatment, there were no statistically significant differences in age, gender, serum biochemical indicators, and other general clinical data among the four groups (all *P* > 0.05), indicating comparability. Specific data are shown in Table 1.

### 3.2. Chest CT Examination

Before treatment, all patients underwent CT examination, and there were no statistical significances in the number, location, and size of pleural tuberculoma among the four groups (all *P* > 0.05), indicating comparability. Specific data are shown in Table 2.

### 3.3. Comparison of Absorption of Lesions at Different Time

After 3 months of treatment, the results showed that the number of significantly absorbed cases and effective cases in group D increased, while the number of invalid cases decreased compared with groups A, B, and C. However, there were no statistical significances in the absorption of lesions among the four groups (*χ*^2^ = 8.272, *P* = 0.507). In addition, pairwise comparison showed no significant difference in the absorption of lesions (*P* > 0.05). After 9 months of treatment, there was no statistically significant difference in the absorption of lesions among the four groups (*χ*^2^ = 8.795, *P* = 0.185), but the absorption of lesions in group D was significantly better than that in group A (*P* < 0.05). Specific data are shown in Table 3 and Figures 1–4.

The article "Clinical Study of Different Treatment Methods for Tuberculous Pleuritis Complicated with Pleural Tuberculoma" was retracted in 2023. Reasons: unreliable results or conclusions; lack of ethics approval or compliance; concerns about the data; concerns about the peer review.

### 3.4. Incidence of Adverse Reactions

During the treatment, the incidence of adverse reactions was 56.67% in group A (*n* = 17), 46.67% (*n* = 14) in group B, 30.00% (*n* = 9) in group C, and 20.00% (*n* = 6) in group D. The difference in the incidence of adverse reactions among the four groups was statistically significant (*χ*^2^ = 8.779, *P* = 0.032). Pairwise comparison showed that the incidence of adverse reactions in groups C and D was significantly lower than that in group A (*P* < 0.05). Specific data are shown in Table 4.

### 3.5. Actual Course of Treatment and Outcome

In group A, 19 patients maintained the original antituberculosis chemotherapy regimen, 7 patients adjusted the chemotherapy regimen and extended the treatment time due to adverse drug reactions, and 3 patients were transferred to other hospitals for surgical treatment after 9 months of treatment and continued antituberculosis chemotherapy after surgery. CT follow-up revealed significant absorption of lesions in 18 patients, effective absorption of lesions in 9 patients with improved clinical symptoms, and no significant absorption of lesions in 3 patients. The total course of treatment in group A was 9-22 months, and 10 cases (33.33%) still had residual lesions or pleural thickening at the end of the course. In group B, 26 patients continued the original treatment regimen, and 4 patients had drug withdrawal after significant pleural tuberculoma reduction. CT follow-up showed no significant change in the size and morphology of the lesions after drug withdrawal. In the end, 21 patients had the lesions significantly absorbed, while the remaining cases had lesions significantly reduced and the clinical symptoms improved. The total course of treatment in group B was 9-18 months, and 7 cases (23.33%) still had residual lesions or pleural thickening at the end of the course. In group C, 22 patients continued the original treatment regimen, and 5 patients received aminoglycoside injection on the basis of the original regimen for 2-3 months. CT follow-up showed significant pleural tuberculoma absorption in 20 patients, significant pleural tuberculoma reduction in 7 patients, and insignificant pleural tuberculoma absorption in 3 patients. The total course of treatment in group C was 9-16 months, and 8 cases (26.67%) still had residual lesions or pleural thickening at the end of the course. In group D, 28 patients continued the original treatment plan, and 2 patients stopped taking the drugs after the pleural tuberculoma shrank significantly. CT follow-up showed that the lesions were significantly absorbed in 27 patients and significantly reduced in 3 patients. The total course of treatment in group D was 9-16 months, and there were still 2 cases of residual lesions (6.67%) at the end of the treatment course.

The article "Clinical Study of Different Treatment Methods for Tuberculous Pleuritis Complicated with Pleural Tuberculoma" was retracted in 2023. Reasons: unreliable results or conclusions; lack of ethics approval or compliance; concerns about the data; concerns about the peer review.

## 4. Discussion

Pleural tuberculoma is common in the clinical treatment and follow-up of patients with tuberculous pleuritis, and a few patients have no clear history. Although pleural tuberculoma is a benign proliferative lesion, the lung can be extensively involved. Without active treatment, some lesions will continue to grow and increase in number, which seriously affects the prognosis of the disease [16]. At present, there is no unified treatment standard, and most patients have a good prognosis by extending the course of antituberculosis treatment and increasing the combination of drugs, local injection, or surgery [9, 17].

As antituberculosis drugs are difficult to penetrate in the focus, intrapleural injection of drugs on the basis of systemic antituberculosis treatment can speed up the killing of tuberculosis bacteria and shorten the course of disease [18, 19]. In addition, antituberculosis drugs have much toxic and side effects, so it is of great significance to reduce adverse reactions to improve curative effect and relieve patients' pain. Isoniazid is relatively safe among antituberculosis drugs, with few adverse reactions in conventional doses [20]. Rifampicin can cause many adverse reactions, and it mainly interferes with the combination and excretion of bilirubin and glucuronic acid through bile excretion. Patients can have joint pain, rash, PLT reduction, liver function injury, and jaundice [21, 22]. Pyrazinamide can cause arthrodynia, hyperuricemia, hepatotoxicity, and gastrointestinal reactions, which are related to dose to a certain extent, but the current conventional dose has relatively few side effects [23, 24]. The main adverse effects of ethambutol are blurred vision, eye pain, red-green color blindness, or any vision loss [25]. Rifabutin is generally well tolerated, with interruptions due to rash, gastrointestinal reactions, neutropenia, and occasionally thrombocytopenia [26].

In order to reduce complications and improve efficacy, different treatment regimens were adopted for the four groups of patients in this study. Isoniazid, pyrazinamide, and ethambutol were all given in the same dose in group A and group C. The difference was that rifampicin was used in the antituberculosis regimen in group A, while rifabutin was used in group C. Both rifampicin and rifabutin are commonly used antituberculosis drugs. A number of clinical studies have shown that rifabutin has a stronger antituberculosis effect at the same dose [27], and rifabutin also has a strong activity against strains resistant to rifampicin [28, 29]. In addition, rifabutin also has a higher lipid solubility than rifampicin and can be distributed in tissues of patients for a longer time and at a higher concentration [30]. In this study, the absorption of lesions in group C was slightly better than that in group A at different time, but the difference was not statistically significant (*P* > 0.05), possibly due to the small sample size of this study. Group B and group D were injected with isoniazid in pleural cavity on the basis of antituberculosis drug therapy. Isoniazid is the preferred antituberculosis drug. By injecting isoniazid into the thorax, the chemotherapy drug can directly reach the interior of the lesion, and the high local drug concentration can cause tuberculoma tissue necrosis, liquefication, tumor shrinkage, or even disappearance, improving the efficacy [31, 32]. In this study, the number of significantly absorbed cases and effective cases in group D increased, while the number of invalid cases decreased after 3 months of treatment, but there was no statistical significance in the absorption of lesions among the four groups (all *P* > 0.05). After 9 months of treatment, the absorption of lesions in group D was significantly better than that in group A (*P* < 0.05). These results indicated that HZE+rifabutin+pleural infusion antituberculosis regimen had better clinical efficacy than classical HRZE regimen in the treatment of pleural tuberculoma, which is consistent with the results of literature review. During treatment, the incidence of adverse reactions in the four groups was significantly different (*P* < 0.05), and the incidence of adverse reactions in groups C and D was significantly lower than that in group A (*P* < 0.05). These results indicated that adjusting medication regimen and replacing rifabutin with less toxic and side effects could significantly improve patients' discomfort during treatment.

The article "Clinical Study of Different Treatment Methods for Tuberculous Pleuritis Complicated with Pleural Tuberculoma" was retracted in 2023. Reasons: unreliable results or conclusions; lack of ethics approval or compliance; concerns about the data; concerns about the peer review.

In conclusion, among the four antituberculosis schemes in this study, the clinical efficacy of HZE+rifabutin+pleural infusion regimen is superior to the classical HRZE scheme, with high safety. However, the number of treatment groups in this study was relatively small, and no significant differences were observed in some results between groups. And in the course of treatment, some patients received surgical treatment, some received aminoglycoside injections for 2 to 3 months, and many patients were lost to follow-up. These would affect the research results seriously. Therefore, a large sample and multicenter study is needed to verify the accuracy of the results of this study.

## Figures and Tables

**Figure 1:** Zhao, male, 39 years old. Chest CT plain scan showed a high-density shadow on the right lung. Group A classical HRZE program was adopted. (a) Lesion 20 × 15 mm before treatment (December 16, 2019). (b) The lesion was reduced to 19 × 13 mm after 3 months of treatment (2020.3.24). (c) At the end of treatment (2021.9.13), the lesion was obviously absorbed, but there was still a residual of 14 × 10 mm.

**Figure 2:** Zhang, male, 32 years old. Chest CT plain scan showed a high-density shadow in the left lung. Group B HRZE+pleural infusion was adopted for treatment. (a) Lesion 28 × 25 mm before treatment (2020.4.29). (b) After 3 months of treatment (2020.7.16), the lesion was reduced to 22 × 20 mm. (c) At the end of treatment (2021.7.7), the lesions were significantly absorbed.

**Figure 3:** Liu, male, 42 years old. Chest CT plain scan showed two high-density shadows in the right lung, which was treated with group C HZE+rifabutin regimen. (a) Before treatment (2020.9.28), the lesion was 30 × 22 mm. (b) After 1 month of treatment (2020.11.02), the lesion was reduced to 22 × 20 mm. (c) After 5 months of treatment (2021.2.6), the lesion was reduced to 18 × 16 mm.

**Figure 4:** Wang, male, 47 years old. Chest CT plain scan showed a high-density shadow in the left lung. Group D HZE+rifabutin+pleural infusion was adopted for treatment. (a) The lesion was 25 × 18 mm before treatment (2020.9.8). (b) After 3 months of treatment (2020.11.23), the lesion was reduced to 22 × 13 mm. (c) The lesions were significantly absorbed after 7 months of treatment (2021.3.19).

**Table 1:** Comparison of general clinical data of patients in four groups.

Group	Group A (*n* = 30)	Group B (*n* = 30)	Group C (*n* = 30)	Group D (*n* = 30)	*F/χ* ^2^	*P*
Gender (male/female)	19/11	20/10	22/8	18/12	1.297	0.730
Age (years)	36.26 ± 2.41	37.31 ± 2.16	36.74 ± 2.48	37.15 ± 2.71	1.949	0.126
Alb (g/L)	37.15 ± 2.34	37.68 ± 2.44	37.43 ± 2.25	37.51 ± 2.27	1.729	0.165
ESR (mm/60 min)	18.41 ± 1.67	19.05 ± 2.10	18.57 ± 2.03	18.79 ± 1.68	0.619	0.604
BG (mmol/L)	5.92 ± 2.16	5.78 ± 2.45	5.69 ± 2.37	5.81 ± 2.43	0.855	0.467
LDH (U/L)	178.26 ± 15.30	176.52 ± 12.47	180.28 ± 14.61	179.04 ± 11.59	0.716	0.544
Complication						
Tuberculous pleuritis	30	30	30	30	—	—
Secondary pulmonary tuberculosis	12	7	15	10	4.8980	0.181
Duration of PTM					1.015	0.985
Less than 3 months	11	13	10	12		
3~6 months	13	13	14	13		
More than 6 months	6	4	6	5		

Note: group A: classical HRZE scheme; group B: HRZE+pleural cavity infusion; group C: HZE+rifabutin; group D: HZE+rifabutin+pleural cavity infusion.

The article "Clinical Study of Different Treatment Methods for Tuberculous Pleuritis Complicated with Pleural Tuberculoma" was retracted in 2023. Reasons: unreliable results or conclusions; lack of ethics approval or compliance; concerns about the data; concerns about the peer review.

**Table 2:** Comparison of CT examination results among four groups.

Group	Group A (*n* = 30)	Group B (*n* = 30)	Group C (*n* = 30)	Group D (*n* = 30)	*χ* ^2^	*P*
Number of pleural tuberculoma	37	40	38	35	—	—
Single lesion	23	22	24	21	0.889	0.828
Multiple lesions	7	8	6	9		
Pleural tuberculoma site					1.562	1.000
Right anterior chest wall	5	5	4	4		
Left anterior chest wall	2	3	2	2		
Right chest wall	3	4	3	3		
Left chest wall	3	5	5	4		
Right posterior chest wall	16	17	15	16		
Left posterior chest wall	8	6	7	6		
Pleural tuberculoma size (mm)	18.2 × 40.3 40.6 × 25.1	18.6 × 39.5 41.5 × 58.4	17.8 × 41.2 38.6 × 67.2	19.5 × 40.5 41.0 × 64.7	—	—

Note: group A: classical HRZE scheme; group B: HRZE+pleural cavity infusion; group C: HZE+rifabutin; group D: HZE+rifabutin+pleural cavity infusion.

**Table 3:** Comparison of absorption of lesions in four groups (*n*, %).

Group	Time	Significant absorbed	Effective	Invalid	Deteriorated
Group A (*n* = 30)	3 months	5 (16.67)	13 (43.33)	11 (36.67)	1 (3.33)
	9 months	12 (40.00)	10 (33.33)	8 (26.67)	0
Group B (*n* = 30)	3 months	8 (26.67)	14 (46.67)	8 (26.67)	0
	9 months	14 (46.67)	10 (33.33)	6 (20.00)	0
Group C (*n* = 30)	3 months	6 (20.00)	15 (50.00)	9 (30.00)	0
	9 months	13 (43.33)	9 (30.00)	8 (26.67)	0
Group D (*n* = 30)	3 months	9 (30.00)	17 (57.67)	4 (15.26)	0
	9 months	22 (73.33)	5 (16.67)	3 (10.00)	0

Note: group A: classical HRZE scheme; group B: HRZE+pleural cavity infusion; group C: HZE+rifabutin; group D: HZE+rifabutin+pleural cavity infusion. *χ*^2^_A−B:3_ = 2.203, *P*_A−B:3_ = 0.531; *χ*^2^_A−C:3_ = 1.434, *P*_A−C:3_ = 0.698; *χ*^2^_A−D:3_ = 5.943, *P*_A−D:3_ = 0.114; *χ*^2^_B−C:3_ = 0.379, *P*_B−C:3_ = 0.827; *χ*^2^_B−D:3_ = 1.682, *P*_B−D:3_ = 0.431; *χ*^2^_C−D:3_ = 2.648, *P*_C−D:3_ = 0.266; *χ*^2^_A−B:9_ = 0.440, *P*_A−B:9_ = 0.803; *χ*^2^_A−C:9_ = 0.093, *P*_A−C:9_ = 0.955; *χ*^2^_A−D:9_ = 6.881, *P*_A−D:9_ = 0.032; *χ*^2^_B−C:9_ = 0.375, *P*_B−C:9_ = 0.829; *χ*^2^_B−D:9_ = 4.444, *P*_B−D:9_ = 0.108; *χ*^2^_C−D:9_ = 5.730, *P*_C−D:9_ = 0.057.

**Table 4:** Comparison of adverse drug reactions in 4 groups.

Group	Skin rash	PLT decrease	ALT increase	UA increase	Total
Group A (*n* = 30)	6	3	10	8	17
Group B (*n* = 30)	4	5	8	5	14
Group C (*n* = 30)	3	3	6	4	9
Group D (*n* = 30)	4	2	3	4	7

Note: group A: classical HRZE scheme; group B: HRZE+pleural cavity infusion; group C: HZE+rifabutin; group D: HZE+rifabutin+pleural cavity infusion. *χ*^2^_A−B:3_ = 0.601, *P*_A−B:3_ = 0.438; *χ*^2^_A−C:3_ = 4.344, *P*_A−C:3_ = 0.037; *χ*^2^_A−D:3_ = 6.944, *P*_A−D:3_ = 0.008; *χ*^2^_B−C:3_ = 1.763, *P*_B−C:3_ = 0.184; *χ*^2^_B−D:3_ = 3.590, *P*_B−D:3_ = 0.058; *χ*^2^_C−D:3_ = 00.341, *P*_C−D:3_ = 0.559.

The article "Clinical Study of Different Treatment Methods for Tuberculous Pleuritis Complicated with Pleural Tuberculoma" was retracted in 2023. Reasons: unreliable results or conclusions; lack of ethics approval or compliance; concerns about the data; concerns about the peer review.

## Data Availability

The labeled datasets used to support the findings of this study are available from the corresponding author upon request.
